# Deep Learning in Cancer Diagnosis and Prognosis Prediction: A Minireview on Challenges, Recent Trends, and Future Directions

**DOI:** 10.1155/2021/9025470

**Published:** 2021-10-31

**Authors:** Ahsan Bin Tufail, Yong-Kui Ma, Mohammed K. A. Kaabar, Francisco Martínez, A. R. Junejo, Inam Ullah, Rahim Khan

**Affiliations:** ^1^School of Electronics and Information Engineering, Harbin Institute of Technology, Harbin 150001, China; ^2^Department of Electrical and Computer Engineering, COMSATS University Islamabad, Sahiwal Campus, Sahiwal 57000, Pakistan; ^3^Gofa Camp, Near Gofa Industrial College and German Adebabay, Nifas Silk-Lafto, 26649 Addis Ababa, Ethiopia; ^4^Institute of Mathematical Sciences, Faculty of Science, University of Malaya, Kuala Lumpur 50603, Malaysia; ^5^Department of Applied Mathematics and Statistics, Technological University of Cartagena, Cartagena 30203, Spain; ^6^School of Control Science and Control Engineering, Harbin Institute of Technology, Harbin 150001, China; ^7^College of Internet of Things (IoT) Engineering, Hohai University (HHU), Changzhou Campus, 213022, China

## Abstract

Deep learning (DL) is a branch of machine learning and artificial intelligence that has been applied to many areas in different domains such as health care and drug design. Cancer prognosis estimates the ultimate fate of a cancer subject and provides survival estimation of the subjects. An accurate and timely diagnostic and prognostic decision will greatly benefit cancer subjects. DL has emerged as a technology of choice due to the availability of high computational resources. The main components in a standard computer-aided design (CAD) system are preprocessing, feature recognition, extraction and selection, categorization, and performance assessment. Reduction of costs associated with sequencing systems offers a myriad of opportunities for building precise models for cancer diagnosis and prognosis prediction. In this survey, we provided a summary of current works where DL has helped to determine the best models for the cancer diagnosis and prognosis prediction tasks. DL is a generic model requiring minimal data manipulations and achieves better results while working with enormous volumes of data. Aims are to scrutinize the influence of DL systems using histopathology images, present a summary of state-of-the-art DL methods, and give directions to future researchers to refine the existing methods.

## 1. Introduction

Cancer is defined as abnormal cell growth that arises from any body organ. In essence, further growth of the cells in these organs is saturated. These silent and saturated cells are increased at a rapid rate till either their removal through a physical procedure such as surgery, medication, use of hormonal therapy, or radiation therapy or their disappearance on their own naturally. The natural disappearance of cancer cells can happen in cancers related to kidney or melanomas. These cells can be screened using tools such as colonoscopy or pap smear examination or using mammograms. There are more than 150 different kinds of cancer, and there is a lack of strategies to cure them in their early stages. Cancer stem cells are an effective way to form stromal cells thus paving a way for the cure of cancers. Apart from stem cells, WNT16B protein also increases resistance against cancer along with chemotherapy. Therapies such as laser therapy and cryotherapy are some of the most vibrant approaches to treat cancer. Some of the most prevalent types of cancers worldwide include lip, oral cavity, breast and cervical, and thyroid cancers. On the other hand, rare cancers such as osteosarcoma, Ewing's sarcoma, male breast cancer, gastrointestinal stromal tumors, chondrosarcoma, mesothelioma, adrenocortical carcinoma, cholangiocarcinoma, kidney chromophobe carcinoma, pheochromocytoma and paraganglioma, sarcoma, and ependymoma made up more than 20% of cancer cases and are rare types of cancers [1–4].

Cancer is a disease of genes. The process of replication, mitosis, and bombardment by oxygen cells bring continuous changes in normal and cancer cells. This process begins at the birth of a cancer cell and goes on till death. During this process, cancer cell gains mass using stromal support cells, immune cells, and endothelial cells. These cells become a part of cancer mass due to factors like stress ligands and antigens. Other emblems of cancer-based cellular stress are proteotoxicity, metabolic changes, and displaced acids of nucleotides. Another pattern of genes that drive them is chromosomes. They are drivers of a cell's nucleus. The human body has around 20,000 genes in somatic cells, and their study known as cytogenetics has seen large strides of progress over the past several decades where it is now possible to build a 3D model of chromosomes [5–7].

Sugar is an important constituent of tumor cells that fuels the rapid growth of these cells. They are an important part of the diet of cancer cells, and their growth ensures the formation of new clones. Bacteria and microbial cells colonize the human body. Microbial cells are estimated to be as abundant as human cells, yet their genome is roughly 100 times the human genome, providing significantly more genetic diversity. Helicobacter pylori, Chlamydia trachomatis, Salmonella enterica serovar typhi, Fusobacterium nucleatum, enterotoxigenic Bacteroides fragilis, Koribacteraceae, etc., are some of the most prominent bacteria that are associated with cancer. Apoptosis and necroptosis are two avenues of programmed cell death [8–10].

Cancer has long inspired fears. In the distant past, physicians related depression or melancholic humour to cancer's pathogenesis. It was believed that melancholy could give rise to a tumor as people attributed their cancer to sadness. Recently, inflammation and nonspecific immune activation are found to be key factors in the pathophysiology of depression related to cancer. Urban centers are at an increasing risk of cancer-related risks due to factors like nutrition; infections such as sea turtle fibropapillomatosis and feline immunodeficiency virus; urban chemical pollution such as carcinogens, polychlorinated biphenyls, glutathione, and urethane-induced adenomas; light and noise pollution such as suppression of pineal melatonin production; changes in survival; and life history strategies [11–13].

Deep learning (DL) has seen phenomenal growth in recent years in the use of artificial intelligence allowing complex computational models to represent abstractions gathered from data with wide applications in speech processing, visual processing, and other domains. These methods work by discovering fine structures in large and often complex datasets using a backpropagation algorithm. Compared to DL, conventional methods such as machine learning-based methods have limitations in processing natural data in its basic form without preprocessing [14].

Convolutional Neural Networks (CNNs) are DL systems equipped with the power to learn invariant features. CNNs have filter banks, feature pooling layers, batch normalization layers, dropout layers and dense layers that work in harmony to create patterns for different object recognition tasks such as detection, segmentation, and classification. CNNs have multilevel hierarchies where the distribution of inputs changes during the process of training. Preprocessed inputs, such as those obtained through the process of whitening, etc., are highly desirable to obtain better performances across tasks [15]. CNNs have many different variants such as those offering shorter connections, for example, DenseNet architecture, which offer advantages in terms of feature circulation and offer substantial reduction in hyperparameters to build efficient architectures [16]. The focal and nonfocal electroencephalogram signals in tunable *Q*-factor wavelet transform domain have been investigated and identified with the help of feature selection and neural network methods [17]. A recent study concerning the low-density parity-check (LDPC) codes for Internet of things networks has been conducted via a novel technique for obtaining the first two minima of check-node update operation of the min-sum-LDPC decoder [18]. In addition, a review of future robust networks including various scenario for 6G has been discussed in [19].

Other types of CNN architectures that have gained popularity in recent years are ResNets, Xception, and GoogLeNet architectures. The need for these networks arises due to degradation in performances across tasks when the network is getting deeper, the need for multiscale processing, and the search for better architectures with less number of parameters [20–23].

Another issue that holds considerable importance in DL is the ability of an architecture to store information over extended time intervals. One solution proposed for this problem is Long Short-Term Memory (LSTM). LSTM architecture works by enforcing consistent error flow that is nonglobal in space and time through states of specialized units [24].

Another idea worth mentioning in DL is the notion of transfer learning. In transfer learning, features extracted from deep CNNs are repurposed to new and novel tasks. The need arises because generic tasks may differ by a wide margin from the original tasks due to which there may be insufficient labelled or other data to train or adapt a DL architecture to new tasks. Using transfer learning, features can be adapted to have sufficient generalization expression using simple techniques reliably [25–27].

Finding better architecture design parameters for DL models is a problem worth considering. Reinforcement learning methods can help in this task. An inspirational example is NASNet architecture that uses a number of different network topologies to find repeated motifs that can be combined in series to handle inputs of varying spatial dimensions and depth [28, 29].

This paper presents an overview of DL methods for the task of cancer diagnosis, prognosis, and prediction. The aim is to highlight the differences between different model constructions and to provide limitations and future perspectives for further exploration of this exciting domain.

The rest of the paper is organized as follows.  Section 2 presents the gist behind the selection of studies that are made a part of this survey article.  Section 3 presents an overview of publically available datasets for cancer research followed by the description of current applications of DL in cancer diagnosis, prognosis, and prediction tasks in Section 4.  Section 5 presents the discussion covering limitations of the existing methods, perspectives, and some directions for future work. Finally, Section 6 concludes this work and proposes avenues for further research in this domain.

## 2. Methodology

The criterion used for the selection of articles for this minireview was language and authenticity of electronic sources. Articles written only in English language are made a part of this survey due to wide recognition of English as the language of scientific and biomedical domains. Years of sources of articles considered for this study range between 1997 and 2020. We used PubMed, Web of Science, IEEE Xplore, and Science Direct platforms to conduct the research. The search terms used were diagnosis of cancer, prognosis of cancer, prediction of cancer using DL, and transfer learning models.

## 3. Publically Available Datasets for Cancer Research Using DL Methods

In this section, we will provide a brief description of publically available datasets for cancer studies. We will briefly describe The Cancer Genome Atlas (TCGA) database, Rotterdam tumor bank, Study to Understand Prognoses and Preferences for Outcomes and Risks of Treatment (SUPPORT), Molecular Taxonomy of Breast Cancer International Consortium (METABRIC), MITOS-ATYPIA-14 dataset, Tumor Proliferation Assessment Challenge (TUPAC) 2016 dataset, INbreast database, Lung Image Database Consortium and Image Database Resource Initiative (LIDC-IDRI) datasets, Lung Nodule Analysis (LUNA16) dataset, Breast Cancer Histopathological Image Classification (BreakHis) dataset, 2015 Bioimaging breast histology classification challenge, Cancer Metastases in Lymph Nodes Challenge breast cancer metastasis detection (CAMELYON) dataset, PatchCamelyon dataset, 2018 International Conference on Image Analysis and Recognition (ICIAR) dataset, MITOS12 dataset, Leukemia microarray gene data, Gene Expression Omnibus repository, BioGPS data portal, The Cancer Imaging Archive (TCIA), Genomic Data Commons (GDC), Therapeutically Applicable Research to Generate Effective Treatments (TARGET), 1000 Genomes Project, Kvasir dataset, University of California Santa Barbara Bio Segmentation Benchmark (UCSB-BB) dataset, and the Multimodal Brain Tumor Image Segmentation Benchmark (BRATS) dataset.

1. *TCGA Database*. Beginning in 2006, TCGA is a result of a joint partnership between the National Cancer Institute and the National Human Genome Research Institute characterizing over 20,000 primary cancer and matched normal samples spanning 33 cancer types such as acute myeloid leukemia, adrenocortical carcinoma, breast lobular carcinoma, and uveal melanoma. The total number of cases in this database is approximately 11,125. It also contains cases of rare types of cancers. This database is available at https://www.cancer.gov/about-nci/organization/ccg/research/structural-genomics/tcga (accessed on September 24, 2021).
2. *Rotterdam Tumor Bank*. This dataset [30] is comprised of 2982 primary breast cancer patients of whom 1546 are positive cases, i.e., they had the disease. Different factors such as estrogen receptors, progesterone receptors, hormonal treatment, number of positive lymph nodes, differentiation grade, and tumor size characterize this dataset. An R package of this dataset can be accessed at https://stat.ethz.ch/R-manual/R-devel/library/survival/html/rotterdam.html (accessed on September 24, 2021).
3. *SUPPORT Database*. This database [31], gathered with the support of five teaching hospitals in the United States, is comprised of 9105 adults with an overall 6-month mortality rate of 47%. Subjects are recruited in two phases. Phase I recruited 4301 patients while phase II recruited 4804 patients. In phase II, the intervention group has 2652 subjects while the control group has 2152 subjects. Patients are diagnosed with one of nine life-threatening diagnoses.
4. *METABRIC Dataset*. This dataset [32] is comprised of 2509 primary breast tumor subjects with 548 matched normal subjects. There are 2506 breast cancer subjects and 3 breast sarcoma subjects. Subjects with breast invasive ductal carcinoma are the most frequently occurring in this dataset while subjects of metaplastic breast cancer and breast angiosarcoma are the least frequently occurring classes. In total, there are eight classes of cancer subjects. This dataset is available at https://www.cbioportal.org/study/summary?id=brca_metabric (accessed on September 24, 2021).
5. *MITOS-ATYPIA-14 Dataset*. This dataset contains histological images of breast cancer for the detection of mitotic cells and for the evaluation of nuclear atypia score for the prognosis of breast cancer. These annotations are provided by two senior and three junior pathologists. The dataset provides samples of haematoxylin and eosin-stained slides with the size of 1539 × 1376 pixels at 20x and 40x magnification levels. For every slide, the pathologists selected several frames at ×10 magnification which are further subdivided into four frames at ×20 magnification which are further subdivided into four frames at ×40 magnification. Evaluation metrics for mitosis are the number of detected mitosis, number of true positives, number of false positives, number of false negatives, sensitivity, precision, and *F*_1_-value. This dataset is available at https://mitos-atypia-14.grand-challenge.org/Home/ (accessed on September 24, 2021).
6. *TUPAC 2016 Dataset*. This dataset [33] provides a way to predict tumor proliferation scores from whole-slide images. The challenge dataset is made up of 500 training and 321 testing breast cancer histology whole-brain slides. This dataset is designed to fulfill three purposes. The first one is to predict mitotic scores while the second one is to predict gene expression-based proliferation scores. A third task was later added to the challenge for mitosis detection.
7. *INbreast Dataset*. This breast cancer dataset [34] has a total of 115 cases and is made up of full-field digital mammograms. The number of images of these cases is 410. In these 115 cases, 90 cases are from women with both breasts affected while 25 cases represent mastectomy patients. Several types of lesions such as masses, calcifications, asymmetries, multiple findings, normal, and distortions are included. Eight cases also have images acquired at different timings.
8. *LIDC-IDRI Database*. Initiated by the National Cancer Institute (NCI), this dataset [35] of Computed Tomography (CT) scans contains 1018 cases of three categories: nodule ≥ 3 mm, nodule < 3 mm, and nonnodule ≥ 3 mm. A two-phase image annotation process was performed by four experienced thoracic radiologists. The goal of this dataset is to identify as completely as possible all lung nodules in each CT scan. This dataset is available at https://wiki.cancerimagingarchive.net/display/Public/LIDC-IDRI#1966254194132fe653e4a7db00715f6f775c012 (accessed on September 24, 2021).
9. *LUNA16 Dataset*. Collected from the LIDC-IDRI dataset, the LUNA16 [36] dataset is designed for the detection of pulmonary nodules from CT scans. The scans where slices were thicker than 2.5 mm were excluded. It facilitates lung nodule segmentation by providing the option of multiple candidates per nodule. In total, this dataset includes 888 CT scans. Irrelevant findings that were not made a part of this dataset include nonnodules, nodules < 3 mm, and nodules annotated by only 1 or 2 radiologists. This dataset is available at https://luna16.grand-challenge.org/Data/ (accessed on September 24, 2021).
10. *BreakHis Dataset*. This dataset [37] of breast cancer subjects contains 9109 microscopic images. These images of tumor tissue are collected from 82 subjects at four different magnification levels which are 40x, 100x, 200x, and 400x. It contains 2480 benign and 5429 malignant samples. These samples are stored in PNG format. The resolution of each sample is 700 × 460 pixels, 3-channel RGB with eight-bit depth in each channel. This database resulted from the collaboration of the P&D Laboratory Pathological Anatomy and Cytopathology, Parana, Brazil, and Laboratory of Vision, Robotics, and Imaging, Federal University of Parana, Brazil. Benign tumors are slow-growing and remain localized to a region while malignant tumors can spread to distant regions and possess the ability to destroy adjacent structures which may cause death. This dataset is available at https://web.inf.ufpr.br/vri/databases/breast-cancer-histopathological-database-breakhis/ (accessed on September 24, 2021).
11. *2015 Bioimaging Breast Histology Classification Challenge Dataset*. This dataset [38] of breast cancer subjects has four classes which are normal, benign, in situ carcinoma, and invasive carcinoma. It has high-resolution, uncompressed, and annotated H&E stain slides. The images have a resolution of 2040 × 1536 pixels. It supports both image and patch-wise classification tasks. This dataset is available at https://rdm.inesctec.pt/dataset/nis-2017-003 (accessed on September 24, 2021).
12. *CAMELYON Dataset*. This dataset [39] is designed for breast cancer metastasis detection and classification in whole-slide images of histological lymph nodes. It facilitates patient-level analysis by combining the assessment of several lymph node slides into one outcome for direct deployment in a clinical setting which will facilitate pathologists while at the same time reducing the subjectivity in diagnosis. It contains 1399 unique whole-slide images of lymph nodes which have a slide-level label indicating whether it contains no metastases, macrometastases, micrometastases, or isolated tumor cells. In addition, the dataset has detailed contours drawn by experts for all metastases in 209 whole-slide images. This dataset is available at https://camelyon17.grand-challenge.org (accessed on September 24, 2021).
13. *PatchCamelyon Dataset*. This dataset [40] contains histopathologic scans of breast cancer lymph node sections. Each image in this dataset is annotated with a label to indicate the presence of metastatic tissue. It contains 327,680 color images with a resolution of 96 × 96 pixels. It is trainable on a single GPU. For size comparisons, it is bigger than CIFAR10 and smaller than the ImageNet dataset. This dataset is available at https://www.tensorflow.org/datasets/catalog/patch_camelyon (accessed on September 24, 2021).
14. *2018 ICIAR Dataset*. This dataset is composed of haematoxylin and eosin-stained breast histology microscopy and whole-slide images. The images are labelled as normal, benign, in situ carcinoma, or invasive carcinoma. There are a total of 400 microscopy images with 100 images per class stored with .tiff extension. The microscopy images are color images with a dimension of 2048 × 1536 pixels. The whole-slide images are color images with a dimension of 42113 × 62625 pixels and are stored in .svs format with pixel-wise labels. This dataset is available at https://iciar2018-challenge.grand-challenge.org/Dataset/ (accessed on September 24, 2021).
15. *MITOS12 Dataset*. This dataset [41] contains 50 breast cancer biopsy slides at a 40x magnification level with more than 300 mitoses in these slides. The dimensions of these images are 2084 × 2084 pixels and 2252 × 2250 pixels. This dataset is helpful with mitotic count to estimate the aggressiveness of the breast tumor. This dataset is available at http://ludo17.free.fr/mitos_2012/dataset.html (accessed on September 24, 2021).
16. *Leukemia Microarray Gene Data*. This dataset [42] contains gene expression data from 60 bone marrow samples of patients belonging to acute lymphoblastic leukemia, acute myeloid leukemia, chronic lymphocytic leukemia, chronic myeloid leukemia, and healthy bone marrow. Microarray technology has been instrumental in genome-wide expression studies especially as the knowledge of metazoan genomes is improving. Further information about this dataset is available at https://www.bioconductor.org/packages/devel/data/experiment/manuals/leukemiasEset/man/leukemiasEset.pdf (accessed on September 24, 2021).
17. *Gene Expression Omnibus Repository*. This repository [43] provides comprehensive sets of microarray, next-generation sequencing, and other genomic data to facilitate research in different types of cancers. Further information about this repository is available at https://www.ncbi.nlm.nih.gov/geo/ (accessed on September 24, 2021).
18. *BioGPS Data Portal*. This portal [44] supports eight species which are humans, mouse, rat, fruitfly, nematode, zebrafish, thale-cress, frog, and pig to facilitate research in genes. Many different kinds of cancers are supported such as lung cancer, breast cancer, esophageal cancer, thyroid cancer, pancreatic cancer, colorectal cancer, and colon cancer. This portal is available at http://biogps.org/#goto=welcome (accessed on September 24, 2021).
19. *TCIA*. This service [45] provides deidentification and hosting of a large archive of medical images of cancer for public access using different modalities such as Magnetic Resonance Imaging (MRI), CT, and digital histopathology. It also provides supporting data such as patient outcomes, treatment details, and genomics. This service is available at https://www.cancerimagingarchive.net (accessed on September 24, 2021).
20. *GDC*. This portal provides genomic, clinical, and biospecimen data for different types of cancers such as bone marrow, breast, eye, skin, lung, liver, and nervous system. It supports cancer research initiatives such as TCGA and TARGET. This portal is available at https://gdc.cancer.gov (accessed on September 24, 2021).
21. *TARGET*. This program provides vast amounts of genomic data to estimate molecular alterations in childhood cancers. The goal is to use data for the development of effective, less toxic therapies. It drives research in acute lymphoblastic leukemia, acute myeloid leukemia, kidney tumors, neuroblastoma, osteosarcoma, etc. Further information is available at https://ocg.cancer.gov/programs/target# (accessed on September 24, 2021).
22. *1000 Genomes Project*. The aim of this project [46] is to find common genetic variants by taking advantage of developments in sequencing technology. It helps in sequencing a large number of people to provide a comprehensive resource on human genetic variation. Cell lines and DNA are available for all 1000 Genomes samples. These samples are completely anonymous with no associated medical data. Further information about this project is available at https://www.internationalgenome.org/1000-genomes-summary (accessed on September 24, 2021).
23. *Kvasir Dataset*. This dataset [47] is accessible at https://dl.acm.org/do/10.1145/3193289/abs/ (accessed on September 24, 2021). It is designed to facilitate research in gastrointestinal (GI) tract cancer. The initial dataset consists of 4000 annotated images belonging to 8 classes with 500 images per class. The anatomical landmarks are Z-line, pylorus, and cecum, while the pathological finding includes esophagitis, polyps, and ulcerative colitis. Resolution of images ranges from 720 × 576 up to 1920 × 1072 pixels. This dataset continues to play an important role in deep learning research.
24. *UCSB-BB Dataset*. This dataset [48] contains images of human, monkey, and cat species at subcellular, cellular, and tissue levels with resolutions ranging from 300 × 200 to 1024 × 1024 pixels. There are 58 images of breast cancer belonging to malignant/benign classes in humans with sizes of 896 × 768 and 768 × 512 at the cellular level associated with ground truth data. This dataset is available at https://bioimage.ucsb.edu/research/bio-segmentation (accessed on September 24, 2021).
25. *BRATS Dataset*. This dataset [49] is composed of clinical and synthetic images. The clinical data has 65 MRI scans of low- and high-grade glioma patients. Four MRI contrasts which are T1, T1c, T2, and FLAIR are represented by clinical data. The synthetic data has 35 high-grade and 30 low-grade glioma subjects. It is aimed at facilitating segmentation of tumors and patient survival through prediction and differentiation between tumor recurrence and progression. This dataset is available at https://www.med.upenn.edu/cbica/brats2020/ (accessed on September 24, 2021).

Table 1 displays a summary of the databases/services/projects to facilitate cancer research covered in this section.

## 4. Current Applications of Deep Learning in Cancer Diagnosis, Prognosis, and Prediction

In this section, we will discuss some current research trends in the domain of DL for cancer diagnosis, prognosis, and prediction tasks. We will cover techniques for the prognosis/prediction of tumors, breast cancer, and other types of cancer. In addition, we will also cover techniques for the segmentation/detection of breast cancer and other types of cancer. Furthermore, we will cover different methods for the classification of breast cancer and other types of cancer. We will also cover techniques for the classification, segmentation, and detection of brain tumors.  Figure 1 shows histopathological views of some of the cancer subtypes that will be covered in this review article.

### 4.1. Prognosis/Prediction of Tumors, Breast Cancer, Skin Cancer, Head and Neck Cancer, Brain Cancer, Liver Cancer, Colorectal Cancer, Ovarian Cancer, and Other Types of Cancer

Petalidis et al. [50] reported a gene expression dataset for astrocytic tumors. They employed an Artificial Neural Network (ANN) algorithm to combine signatures from histopathological subclasses of these tumors in order to address the need for proper grading of these tumors. In this study, they found 59 genes which belong to three classes, namely, angiogenesis, lower-grade astrocytic tumor discrimination, and cell differentiation. They further report that these tumor subtypes have very high prognostic value, and they are missing in other studies reported in the literature. Finally, they report 11 classifiers that used genes to differentiate among primary/secondary subtypes of glioblastomas. They used a custom as well as independent dataset reporting accuracy of 96.15% to identify correct classes for these subtypes. Chi et al. [51] use morphometric features to compare prediction outcomes on two different breast cancer datasets. They report successful predictions with good and bad prognostic values. Here, good means that prognosis stands valuable even after five years while bad suggests less than five years. The authors in [52] conducted experiments in female breast carcinoma patients using a DL approach. They did prediction using a Cox regression model and gene expression datasets. They called their approach Survival Analysis Learning with MultiOmics Neural Networks (SALMON). They report that performance of SALMON is improved when more data is used to combine and simplify cancer biomarkers and gene expressions to enable prognosis prediction. Shimizu and Nakayama [53] conducted experiments to identify breast cancer genes for prognosis prediction using The Cancer Genome Atlas (TCGA) database. They identified 184 genes using artificial intelligence (AI), and for that purpose, they used random forest and neural network models. Furthermore, they used a molecular score for prognosis that uses only 23 of these genes. They confirmed that they have found potential drug targets in these genetic discoveries. The authors in [54] performed their experiments using malignant melanoma. They used a dataset with 1160 females and 786 males. They used an ANN architecture employing a flexible nonlinear structure for prognosis prediction of survival probabilities. They found the performance of their model to be at par with the Cox model with the advantage that it offers a flexible approach when analyzing data using a specified distributional form. Jing et al. [55] introduced a loss function combining a pairwise ranking loss and a mean squared error loss to optimize a DL model validated on four publically available datasets, such as the Worcester Heart Attack Study (WHAS), Rotterdam tumor bank, Study to Understand Prognoses and Preferences for Outcomes and Risks of Treatment (SUPPORT), and Molecular Taxonomy of Breast Cancer International Consortium (METABRIC). Their model achieved superior performance results than medical experts for nasopharyngeal carcinoma prognosis. Hao et al. [56] proposed a DL network predicting prognoses and describing complex biological pathways thus providing their model the power to interpret its outcomes. They conducted experiments for prediction in glioblastoma multiforme brain cancer from TCGA database. Their model achieves an Area under the Curve (AUC) of 0.6622 ± 0.013 and an *F*_1_ score of 0.3978 ± 0.016 outperforming other models such as Logistic Least Absolute Shrinkage and Selection Operator (LASSO), Random LASSO, Support Vector Machines (SVMs), and a dropout neural network model which shows the superiority of their approach. The authors [57] put forward a multimodal DL network integrating multidimensional data. Their model combined gene expression data, alteration data, and other forms of clinical data achieving better performance than models with 1D data and other approaches. Chaudhary et al. [58] proposed the DL-based approach based on a combination of RNA and methylation data from TCGA to model hepatocellular carcinoma subjects. Their model achieves a concordance index of 0.68 and a *p* value of 7.13 × 10^−6^. They found that TP53 mutations, KRT19 and EPCAM stemness markers, and Wnt and Akt signaling pathways are associated with more aggressive subtypes. The authors in [59] proposed a DL model combining CNN and Recurrent Neural Network (RNN) architectures for the prediction of colorectal cancer subjects using digitized haematoxylin-eosin-stained tumor tissue microarray samples. In the low- and high-risk patients, their model achieved a hazard ratio of 2.3 for visual assessment of histological tissues and a hazard ratio of 1.65 on the whole-slide level for both low- and high-risk subjects. Wang et al. [60] come up with a DL model to predict serous ovarian cancer subjects by extracting prognostic biomarkers from CT images. They further proposed a combined DL and Cox hazards model and achieved a concordance index of 0.713 and 0.694 for individual and three years of recurrence probability of subjects, respectively. The authors in [61] used a DL-based ANN model from transcriptomics data. They deployed TCGA datasets of RNA sequences belonging to ten different kinds of cancers. Their model achieved superior or equal level performance at both the pathway and gene levels. The authors in [62] came up with a DL model combining a Cox proportional hazards model with one of the best performing survival methods. They conducted experiments on WHAS, METABRIC, and SUPPORT datasets achieving good prediction performance levels for personalized treatment recommendations. Mobadersany et al. [63] predicted time-to-event results from histopathology images and gene-based biomarkers using CNNs as DL models from glioma and glioblastoma cohorts of TCGA. They used a sampling- and filtering-based approach for the improvement of their predictions by not taking into account the intratumoral heterogeneity. Their model achieved a median concordance index of 0.754 surpassing other state-of-the-art approaches. The authors in [64] developed a DL-based approach using CNNs to predict the survival of mesothelioma cancer subjects. They used TCGA and a French source to test their approach. They achieved a concordance index of 0.656 on the TCGA cohort surpassing the performance of human experts and found key regions in the stroma that are associated with inflammation and cellular diversity. Liu et al. [65] modeled diagnostic prediction using DL models. The authors conducted their study on 27 diverse cancer types obtained from TCGA and Gene Expression Omnibus dataset. They successfully decoded 12 CpG and 13 promoter markers. The CpG markers that they identified achieved a sensitivity of 100% in the prediction of prostate cancer samples while promoter markers achieved 92% using cell-free deoxyribonucleic acid (DNA) methylation data.

Table 2 displays a summary of the studies for the task of prognosis and prediction of cancers covered in this subsection.

### 4.2. Segmentation/Detection of Breast Cancer, Lung Cancer, Bladder Cancer, and Other Types of Cancer

Yap et al. [66] used DL approaches for breast lesion detection using ultrasound images. They investigated the performance of LeNet, U-Net, and a pretrained AlexNet. They conducted their experiments on two custom datasets of 306 and 163 images termed dataset A and dataset B, respectively. Their pretrained AlexNet-based model achieved the best overall performance by achieving an *F*-measure of 0.91 and 0.89 on both datasets. The authors in [67] come up with different variants of fully convolutional networks (FCNs) for the segmentation of lesions of breast cancer subjects. They tried an AlexNet-based FCN, as well as 8-, 16-, and 32-layered FCN models. To overcome the problem of data deficiency, they used transfer learning and pretraining on the ImageNet dataset. Their dataset has two classes, benign and malignant. They reported an average dice score of 0.7626 using FCN with 16 layers on benign lesions. Their model correctly recognized 89.6% of benign lesions and 60.6% of the malignant lesions successfully. Liu et al. [68] used DL to detect breast cancer in lymph node biopsies. They used 399 slides from the Camelyon16 challenge dataset to achieve an AUC of 99% at the slide level. They used a second custom dataset that has 108 slides to achieve an AUC of 99.6%. As a preprocessing step, they used a color normalization procedure. The authors in [69] used different DL methods such as faster region CNN, ResNET-50, and DenseNet-201 architectures for breast cancer detection using histopathology images. They used three datasets to conduct their experiments which are International Conference on Pattern Recognition 2012, MITOS-ATYPIA-14, and Tumor Proliferation Assessment Challenge 2016 dataset. They achieved a precision of 0.876 on the International Conference on Pattern Recognition 2012 dataset, 0.848 on MITOS-ATYPIA-14, and a precision of 0.641 on the Tumor Proliferation Assessment Challenge 2016 dataset. As data augmentation methods, they employed horizontal and vertical flipping, translation, and resizing operations to artificially increase the size of datasets. Anuranjeeta et al. [70] used shape and morphological features derived from segmented images to detect cancer cells using a number of DL and machine learning-based models. They used J-Rip, logistic modal tree, rotation forest, multilayer perceptron, and other models trained by histopathological images. Rotation forest performed the best in cancerous/noncancerous detection achieving an accuracy of 85.7%. The authors in [71] used a modified regional CNN method to efficiently determine mitosis in breast cancer using histopathological images. They employed subjects belonging to the 2014 International Conference on Pattern Recognition (ICPR) and TUPAC 2016 datasets in their study. They achieved 0.76 in precision on the TUPAC 2016 dataset. Zhou et al. [72] used a 3D deep CNN model to detect lesions in the breast cancer MRI dataset. They deployed a custom dataset with 1537 female patients and classify them as benign or malignant. They achieved an accuracy of 83.7% for the diagnostic task and a dice distance score of 0.501 for the detection task. The authors in [73] proposed a DL integrated architecture with the capability of performing classification, segmentation, and detection for the screening of breast masses as benign or malignant. They used digital X-ray mammograms from the INbreast database. Their model achieved a mass detection accuracy of 98.96%, while for mass segmentations, they achieved a dice score of 92.69%. To augment the dataset, the authors applied rotation 8 times to synthetically increase the size of the dataset. Nasrullah et al. [74] deployed DL-based architectures for the diagnosis of malignant nodules in lung cancer. They conducted studies on LUNA16 and LIDC-IDRI datasets. They used faster region CNN and U-Net styled architecture to achieve an accuracy of 94.17% on the classification task. The authors in [75] used a DL-based system for screening lung cancer using CT scans. They used LIDC-IDRI and Kaggle data science bowl challenge datasets for the experiments. Their system was based on 3D CNN architectures. The authors used heavy augmentations to artificially increase the size of the datasets using methods such as rotations, scaling, translation, and reflection. They achieved a dice coefficient of 0.4 on the LIDC-IDRI dataset. Shkolyar et al. [76] deployed DL-based models for the detection of papillary and flat bladder cancer. They used CNNs to construct an image analysis platform. They used two datasets of 100 and 54 subjects. Their model successfully detected 42 of 44 papillary and flat bladder cancers. They reported a per-tumor sensitivity of 90.9%. Fourcade et al. [77] used a combination of DL and superpixel segmentation-based methods to segment full body organs such as the brain and heart from Positron Emission Tomography (PET) images. To synthetically increase the size of the dataset, the authors deployed rotations, scaling, mirroring, and elastic deformations. Their best performing model achieved a dice score of 0.93. The authors in [78] deployed DL architectures to detect brain metastasis on MRI. They used data from 121 subjects in their proposed study. They used a faster region CNN model achieving an area under the ROC curve of 0.79. Ma et al. [79] used you only look once v3 dense multireceptive fields CNN for thyroid cancer nodule detection. They used ultrasound images and deployed different data augmentation methods such as color jitter, change saturation, exposure, and hue on two datasets of 152 and 699 images. The number of images increased to 10845 after the application of data augmentation schemes. The values of mean average precision (mAP) reported by the authors were 90.05 and 95.23. Das et al. [80] proposed a system combining watershed segmentation, Gaussian mixture model (GMM), and deep neural network for the classification and segmentation of liver cancer using CT scans. Their model performed recognition of hemangioma, hepatocellular carcinoma, and metastatic carcinoma subjects. They employed 225 CT scans in their study achieving a dice score of 0.9743 on the testing set for the segmentation task and an accuracy of 99.38% for the multiclass classification task. The authors in [81] proposed a DL-based model for the segmentation of histopathology images of the liver organ. Their proposed DL model combined residual block, bottleneck block, and an attention decoder block. The authors further created a new dataset of 80 histopathology images which they named as the KMC liver dataset and proposed a joint loss function combining dice and Jaccard losses. They conducted their experiments on two datasets: KMC liver and multiorgan Kumar datasets. Each image in the Kumar dataset has a dimension of 1000 × 1000 while each image in the KMC liver dataset has a dimension of 1920 × 1440. Their model achieved a Jaccard index of 0.7206 on the KMC liver dataset and 0.6888 on the Kumar dataset. Wang and Chung [82] proposed a modified U-Net-based architecture for the segmentation and diagnosis of the colon gland. The authors employed two datasets for the experiments: the gland segmentation dataset from Medical Image Computing and Computer-Assisted Intervention (MICCAI) challenge and an independent colorectal adenocarcinoma gland dataset. The authors conducted validation experiments on 378 images augmented using elastic transformation, cropping, rotation, flipping, blurring, and distortion operations. Their model achieved a dice score of 0.929 on the gland segmentation dataset from MICCAI and 0.89 on the independent colorectal adenocarcinoma gland dataset for the segmentation task. The authors in [83] proposed a CNN architecture combining three CNNs for the segmentation and classification of colorectal cancer using MRI images of 28 adenocarcinomas and 5 mucinous carcinomas. Their model achieved a dice score of 0.60, precision of 0.76, and recall of 0.55 on the testing set. The authors used cropping and min–max scaling as preprocessing methods. Juebin et al. [84] proposed segmentation algorithms based on U-Net models from ultrasound images of ovarian cancer. Image clipping was used as a preprocessing method. The methods are validated on 127 patients and a total of 469 images. Their best model achieved a dice score of 0.87, an average Pearson correlation of 0.90, and an average intraclass correlation of 0.89. Shibata et al. [85] used the mask R-CNN algorithm for the segmentation of 1208 healthy and 533 gastric cancer endoscopic images. The resolution of the images ranges from 640 × 480 to 1440 × 1080 pixels. Their model achieved an average dice index of 71%. Wang and Liu [86] proposed an architecture based on Deeplab v3+ for the segmentation of 1340 pathological slices of gastric cancer. The authors used image mirroring, random flip, scale, and rotation as augmentation techniques. Mean subtraction followed by division with variance was used as a preprocessing method. Their model achieved a dice score of 0.9166. Shrestha et al. [87] proposed a DL system combining four U-Net models. They used MRI images of prostate cancer from an online database. Each image has a resolution of 256∗256 pixels. They used a combination of modified dice and binary cross-entropy loss for the segmentation task. They preprocess the images using denoising and intensity normalization procedures achieving an overall average accuracy of 95.3%. Liu et al. [88] proposed a DL method integrating mask R-CNN and Inception version 3 models for the classification, segmentation, and detection tasks of prostate cancer. They used a dataset of 1200 ultrasound images. Their model achieved a dice score of 0.88 and a precision of 76% on malignant and 75% on benign classes for the classification task using an Inception v3 architecture. The authors in [89] proposed a 2D U-Net model deploying CT images of 556 cases of prostate cancer. They achieved a dice score of 0.85, 0.94, and 0.85 for three organs, namely, prostate, bladder, and rectum, respectively. Liang et al. [90] developed a DL-based model employing CNN architecture for the segmentation of pancreatic tumors. The authors deployed a dataset of T1w MRI images of 40 subjects. They achieved a dice score of 0.73 using rotation and flipping as data augmentation methods. The authors in [91] proposed a DL method using spiral transformation to perform segmentation of MRI images of pancreatic cancer. The authors used rotation and spiral transformation as data augmentation methods. They deployed a dataset of MRI images belonging to 73 patients. Their architecture is a combination of ResNet and U-Net architectures. They achieved a dice score of 0.656 ± 0.1021.

Table 3 displays a summary of the studies for the task of segmentation and detection of cancers covered in this subsection.

### 4.3. Classification of Breast Cancer

Huynh et al. [92] used DL methods to classify regions of interest taken from ultrasound images. Cystic, benign, or malignant labels were assigned to each region. Two binary classification tasks were performed using pretrained CNNs, nonmalignant (benign+cystic)/malignant and benign/malignant. They used SVM as a classifier on the CNN-derived features. On the nonmalignant/malignant classification task, they obtained an AUC of 0.9 while on the benign/malignant task, their method obtained an AUC of 0.88. The authors in [93] used CNNs as their DL approaches and introduced the concept of a matching layer to convert grayscale to red, green, and blue patterns. They used 882 ultrasound images obtained from two publicly available datasets. Using fine-tuning and matching layer, their method approached an AUC of 0.936 on a test set of 150 cases. Byra et al. [94] used DL transfer learning-based approaches such as Inception version 3 and VGG19 architectures on reconstructed B-mode images experiencing a decrease in classification performances. To counter this, they used data augmentation to reconstruct B-mode images achieving better performances on breast ultrasound images. The authors in [95] combined cross-modal and cross-domain transfer learning for the benign/malignant classification task. In comparison to training from scratch and simple fine-tuning, their approach achieved better performance with 97% accuracy on ultrasound images. Hadad et al. [96] deployed cross-modal transfer learning using mammography images achieving an accuracy of 0.93 which is better than cross-domain transfer learning. The authors in [97] presented a study on the use of MRI in screening individuals younger than 40 years confirming the effectiveness of MRI as a modality of choice for such diagnoses. They reported a very high sensitivity around 93% to 100% and low specificity in the range of 37% to 97%. They found MRI to be effective especially after reconstructive surgery. Hu et al. [98] developed a transfer learning methodology using an MRI modality with multiple parameters. They used different sequences such as dynamic contrast-enhanced and a T2-weighted sequence to distinguish benign lesions from malignant. They used image, feature, and classifier fusion methods and achieved an AUC of 0.87 for the feature fusion scheme that statistically outperformed other methods. The authors in [99] proposed a methodology using Inception version 4 and the residual network transfer learning architectures as well as a recurrent CNN architecture on the 2015 Breast Cancer Classification Challenge and BreakHis datasets for binary and multiclass classification tasks. They used rotation, translation, and other data augmentation methods to artificially increase the size of the datasets achieving an accuracy of 97.57 ± 0.89% on multiclass and an accuracy of 97.95 ± 1.07% on binary classification tasks. Bayramoglu et al. [100] used single and multitask CNN architectures to predict malignancy and image magnification levels. Cropping and rotation on the BreakHis dataset were deployed to augment the dataset. They achieved a classification rate of 83.72% for the benign/malignant binary classification task using a single task and an accuracy of 82.13% using multitask CNN architecture. The authors in [101] proposed an approach for progressive combining of weak DL classifiers into a stronger classifier for carcinomas/noncarcinomas binary and normal/benign/in situ/invasive carcinomas multiclass (4 classes) classification tasks. They used BreakHis and 2015 bioimaging breast histology classification challenge datasets. They deployed augmentation methods such as reflection, random cropping, rotation, and translation of an image. They achieved a classification accuracy of 99.5% and 96.9% for binary classification tasks using the 2015 bioimaging breast histology classification challenge database and BreakHis database while for multiclass classification, they achieved 96.4% classification accuracy on the 2015 bioimaging breast histology classification challenge database. Kassani et al. [102] used an ensemble of transfer learning architectures for binary classification of breast cancer. They used VGG19, MobileNet, and DenseNet architectures on four benchmark datasets: BreakHis, PatchCamelyon, 2015 Bioimaging challenge, and 2018 ICIAR datasets. They used flipping, zoom, shear, rotation, etc., as data augmentation methods. They achieved accuracies of 98.13%, 94.64%, 95%, and 83.1% on these datasets. The authors in [103] proposed a DL method for multiclass (8 classes) classification of histopathological images on the BreakHis dataset. Data augmentation methods such as rotation, flipping, sharing, and their combinations were deployed to achieve a correct classification rate of 95.48% on the multiclass classification task. Toğaçar et al. [104] deployed a DL model for multiclass (8 classes) classification of breast histopathological images on the BreakHis dataset. They used convolutional, attention, residual, pooling, and dense blocks along with hypercolumn technique to build their architecture. As data augmentation methods, they used flipping, shifting, change of brightness, and rotation achieving 98.51% accuracy. The authors in [105] used a combination of DenseNet and Xception transfer learning architectures for benign/malignant binary and magnification-specific multiclass classification tasks. They used the BreakHis dataset achieving an accuracy of 99% and 92% on binary and multiclass classification tasks, respectively, while deploying stain normalization for preprocessing of images. Spanhol et al. [106] performed experiments for the binary (benign/malignant tumors) classification task using histology images. They report an accuracy of 90.0 ± 6.7% on images obtained from the BreakHis dataset. The authors in [107] proposed a DL model for the multiclass (8 classes) classification task using histopathological images. They conducted experiments on the BreakHis dataset. For data augmentation, the authors deployed rotation, level/vertical flipping, translation techniques, etc., and their combinations achieving a patient-level accuracy of 94.7 ± 3.6%. Bardou et al. [108] compared CNNs and traditional machine learning techniques such as bag of words and linear coding using SVMs. They deployed BreakHis datasets for both binary and multiclass (8 classes) classification tasks to categorize images into benign/malignant classes and their subclasses. The authors achieved accuracies of 98.33% and 88.23% for binary and multiclass classifications, respectively, using the deployed approaches. The authors in [109] combined four residual networks for binary (benign/malignant) and multiclass classification of histology images using the BreakHis dataset. They achieved an accuracy of 96.25% for the eight-class classification task. The authors deployed rotation, flipping, translation, and color variation augmentation as data enhancing methods while stain normalization as a preprocessing method. Budak et al. [110] used a DL model combining FCN and bi-LSTM architectures on the BreakHis dataset for binary (benign/malignant) classification achieving an accuracy of 96.32%. The authors in [111] used a DL-based model for binary (benign/malignant) classification of histopathological images. They performed experiments on the BreakHis dataset fusing ResNet-18, ResNet-50, and AlexNet architectures using belief theory. They achieved an image-level accuracy of 96.88%. Sudharshan et al. [112] deployed a weakly supervised scheme for the binary classification of benign and malignant tumors using histopathology images. They deployed the BreakHis dataset achieving an accuracy of 92.1% at 40x magnification. An important contribution of their approach is the absence of the need for labelling the images. The authors in [38] deployed CNNs for both binary (carcinoma/noncarcinoma) and multiclass (normal/benign/in situ/invasive) classification tasks. They used the 2015 Bioimaging breast histology classification challenge dataset in their study. Their architectures were able to retrieve information at different scales. For the multiclass classification task, the authors achieved an accuracy of 77.8% while for the binary classification task, they achieved an accuracy of 83.3% using rotation and mirroring as data enhancement methods for both these tasks. Rakhlin et al. [113] deployed different transfer learning architectures using microscopic histological images from the ICIAR 2018 Grand Challenge dataset for binary (carcinomas/noncarcinomas) and multiclass (four classes) classification tasks. They used pretrained ResNet-50, Inception version 3, and VGG16 architectures. They deployed normalization, downscaling, cropping, and color variation as augmentation schemes achieving a correct classification rate of 87.2% for multiclass classification and 93.8% for the binary classification task. The authors in [114] extracted smaller/larger patches using a clustering approach and a CNN (ResNet-50 architecture) at cell and tissue levels deploying the 2015 Bioimaging breast histology classification challenge dataset. For the multiclass (4 classes) classification task, the authors reported accuracy of 88.89% using the proposed approach. The authors deployed stain normalization procedure as a preprocessing method. Shallu and Mehra [115] demonstrated the use of three different transfer learning architectures such as VGG16, VGG19, and ResNet-50 for the classification of histological images on the BreakHis dataset. They deployed rotation as the data enhancement scheme. They found the performance of a fine-tuned VGG16 with logistic regression classifier to be the best achieving an accuracy of 92.6% with this classifier. The authors in [116] deployed CNN, *K* nearest neighbour (KNN), Inception version 3, SVM, and ANN algorithms for the binary (benign/malignant) classification task. They used different schemes for preprocessing and data enhancement such as gray scaling, channel standardization, flipping, rotation, and cropping as well as image segmentation to reach an accuracy of 97% using ANN architecture. Bevilacqua et al. [117] evaluated two different frameworks for binary and multiclass classification of irregular/regular/stellar/no opacity lesions from segmented high-resolution images. They used ANN classifiers with hand-crafted and morphological features for the first framework. For the second framework, they used different CNN models especially a VGG model. They reported accuracy of 84.19% for the first framework on binary and 74.84% on multiclass classification tasks while for the second framework, they obtained an accuracy of 92.02% for binary and multiclass classification tasks. The authors in [118] make a contrast between two machine learning approaches for the multiclass (8 classes) classification task using histopathological images on the BreakHis dataset. The first approach used handcrafted features while the second approach used CNN as a feature extractor. They used VGG16, VGG19, and ResNet-50 as their CNN models. They used rotation, translation, scaling, and flipping as data enhancement methods. The VGG16 model reaches an accuracy of 93.25% at the patient level for the multiclass classification task. Spanhol et al. [119] proposed a DL model that reused a previously trained CNN model on the BreakHis dataset achieving an *F*_1_-score of 90.3 at the subject level. The authors in [120] exploited global covariance information using a matrix power normalization procedure into a simple CNN model. This arrangement can exploit second-order statistical information producing effective representations from histological images. On the BreakHis dataset for the binary (benign/malignant) classification task, they achieved an accuracy of 97.92% at the subject level while employing cropping and flipping operations to enhance the size of the dataset synthetically. Khan et al. [121] used different transfer learning (GoogLeNet, VGGNet, and ResNet) architectures for binary classification of benign/malignant tumor cells while deploying BreakHis and a custom dataset. For data augmentation, scaling, rotation, translation, and color augmentation methods were used by them to achieve a correct classification rate of 97.67%. The authors in [122] introduced an information-based architecture that is designed to exploit clinical information. There are six types of records in their dataset of 100 subjects, such as encounter notes, operation records, pathology notes, radiology notes, progress notes, and discharge summaries. They used fine-tuned transformer models from pretrained bidirectional encoder representations achieving a precision of 0.976 for relation recognition. Naik et al. [123] deployed a DL model to assess estrogen status from whole-slide histopathological images. They used the Australian Breast Cancer Tissue Bank as well as TCGA datasets in their study and further deployed flipping, rotation, color jitter, and cutout regularization as augmentation methods. Their model achieved an AUC of 0.861 on TCGA and an AUC of 0.905 on Australian Breast Cancer Tissue Bank datasets. The authors in [124] compared different DL techniques for the classification of mammograms. They used single as well as 4-model averaging to conduct their experiments on INbreast as well as an independent database. They used different data enhancement techniques such as flipping, rotation, intensity shifting, and zoom. The single model achieved an AUC of 0.88 while 4-model averaging achieved an AUC of 0.91 on the independent database. On the INbreast dataset, the single model achieved an AUC of 0.95 while 4-model averaging achieved an AUC of 0.98. Their study shows the superiority of combining models over a single model.

Table 4 displays a summary of the studies for the classification of breast cancer covered in this subsection.

### 4.4. Classification of Colorectal Cancer, Gastric Cancer, Bladder Cancer, Lung Cancer, Prostate Cancer, Skin Cancer, Liver Cancer, Head and Neck Cancer, Pancreatic Cancer, and Other Types of Cancers

Kather et al. [125] deployed different transfer learning architectures for multiclass (9 classes) classification of colorectal cancer subjects. They used VGG19, AlexNet, SqueezeNet, GoogLeNet, and ResNet-50 models on two datasets of 86 and 25 subjects reaching an accuracy of 98.7% and greater than 94% on them. The authors in [126] deployed a CNN architecture to extract features from Optical Coherence Tomography (OCT) images of colorectal cancer subjects. Their network was trained using 26000 OCT images representing 42 areas achieving an AUC of 0.998. Dong et al. [127] deployed a DL method to exploit information in multiphase CT nomograms in gastric cancer subjects. They used three cohorts to test the effectiveness of their model achieving a discrimination rate of 0.821, 0.797, and 0.822 in the primary, external validation, and international validation cohorts. Woerl et al. [128] deployed a DL method to identify bladder cancer from histomorphological images. They used 2 datasets of 407 and 16 subjects each from TCGA and custom cohorts, respectively, achieving accuracies of 69.91% and 75% on TCGA and custom subsets, respectively. Wang et al. [129] used the idea of weakly supervised learning exploiting image-level labels for the classification of lung cancer images. They used two datasets, one from TCGA and the other is a custom dataset. To enhance the training set, color jittering, translation, flipping, and rotation were used.

Their model successfully achieves an accuracy of 97.3% and an AUC of 85.6% on custom and TCGA datasets. Karimi et al. [130] used a DL method combining three separate CNNs that used different patch sizes for the classification of histopathological images with limited data. They used new data enhancement methods such as elastic deformation and augmentation in the space of learned features for binary classification of cancerous/benign and low-grade–high-grade patches achieving an accuracy of 92% and 86%, respectively, on both binary classification tasks. Dascalu and David [131] used DL architectures for binary classification of benign/malignant cases of skin cancer subjects. They used a skin magnifier with polarized light and an advanced dermoscope to construct their datasets. The authors achieved an F2-score sensitivity of 91.7% and 89.5% respectively for skin magnifier with polarized light and advanced dermoscope images. The authors in [132] used DL techniques to build a skin cancer classification model for binary and multiclass classification of malignant and benign skin tumors. They used Kaohsiung Chang Gung Memorial Hospital and HAM10000 datasets in their study. Their model achieved an accuracy of 85.8% on the HAM10000 dataset for 7-class classification tasks. On the Kaohsiung Chang Gung Memorial Hospital dataset, their model achieved an accuracy of 72.1% for 5-class classification and 89.5% for binary classification tasks. Thomas et al. [133] applied interpretable DL models to classify skin cancers in a histopathological setting. They studied three types of cancers basal cell carcinoma, squamous cell carcinoma, and intraepidermal carcinoma. They deployed a multiclass (12 classes) classification model to achieve accuracies between 93.6% and 97.9%. To solve the class imbalance problem and to increase the size of the dataset, they used flipping and rotation as data augmentation methods to increase the size of the dataset 8 times. The authors in [134] developed a CNN model for the classification of melanoma and nevi. They used a dataset of 11444 images belonging to five categories. They deployed novel DL techniques to train a single CNN model. In addition, they also asked 112 dermatologists to grade the images. Then, they used a gradient boosting method to develop a new classifier for binary (benign/malignant) and multiclass (5 classes) classification tasks achieving accuracies of 86.5% and 82.95% on both these tasks. Sun et al. [135] developed a DL method to classify liver cancer subjects as abnormal/normal on publically available TCGA datasets. Transfer learning and multiple instance learning were combined for the classification of patch features. The authors used tissue extraction, color normalization, and patch extraction for preprocessing of histopathological images. Diao et al. [136] used a transfer learning-based CNN architecture named Inception version 3 to classify nasopharyngeal carcinoma subjects into three classes. They used a total of 1970 images of 731 subjects. The three classes considered in their study were chronic nasopharyngeal inflammation, lymphoid hyperplasia, and nasopharyngeal carcinoma. Their model achieved a mean AUC of 0.936. Liu et al. [137] used a CNN classifier to diagnose subjects with pancreatic cancer using contrast-enhanced CT images. They used three different datasets to test the effectiveness of their approach. The first dataset named local test set 1 has 295 patients with pancreatic cancer and 256 controls for training and 75 patients with pancreatic cancer and 64 controls for validation. The second dataset named local test set 2 has 101 patients with pancreatic cancers and 88 controls while the third dataset named the US dataset has 281 pancreatic cancer subjects and 82 controls. In local test set 1, local test set 2, and US datasets, their model achieved an accuracy of 98.6%, 98.9%, and 83.2%, respectively. To augment the datasets, the authors used moving window and flipping operations. Korfiatis et al. [138] compared the performances of ResNet-18, ResNet-34, and ResNet-50 architectures for the classification of MRI scans of 155 subjects for multiclass (3 classes) classification of no tumor, methylated methylguanine methyltransferase methylation, or nonmethylated classes. ResNet-50 architecture achieved the best performance with an accuracy of 94.9%; ResNet-34 architecture achieved an accuracy of 80.72% while ResNet-18 architecture achieved an accuracy of 76.75%. The authors in [139] used a two-phase training to study and mitigate class biasedness using a DL-based CNN model for the classification of breast cancer histological images. They conducted their experiments using MITOS12 and 2016 Tumor Proliferation Assessment Challenge datasets. Prior to phase 1 of training, segmentation using the global binary thresholding method was applied. In phase 1, a CNN was trained on the segmented patches using rotation and flipping data augmentation methods as well as the blue ratio histogram-based *k*-means clustering approach. In phase 2, the dataset was again modified to reduce the effects of class imbalance yielding an *F*-measure of 0.79. Campanella et al. [140] proposed a DL-based system utilizing information from multiple instances in order to help the pathologists exclude information without compromising performance metrics. They used 44732 whole-slide images belonging to 15187 patients. They achieved AUC above 0.98 and 100% sensitivity for prostate cancer, basal cell carcinoma, and breast cancer metastases to axillary lymph nodes. The authors in [141] proposed two DL-based systems to detect myeloid leukemia from the leukemia microarray genetic dataset. The first DL system is a single-layered neural network while the second one has 3 hidden layers. They used information of 22283 genes extracted from the Gene Expression Omnibus repository. Their models achieved accuracies of 63.33% and 96.67% for single and multilayered DL architectures with a significant normalization test (*p* > 0.05). Jeyaraj and Samuel Nadar [142] used a regression-based DL algorithm to investigate hyperspectral images to diagnose oral cancer. Their system extracted patches for classification into normal, benign, and malignant classes using BioGPS, TCIA, and GDC datasets. For 100 malignant image patch training, they achieved an accuracy of 91.4% while for 500 malignant image patch training, they achieved an accuracy of 94.5%. The authors in [143] proposed a DL method to study the relationship between genomic variations and traits. They analyzed 6083 sample exon sequencing files belonging to 12 cancer types. They used TCGA and 1000 Genomes Project. They performed both binary (cancer/healthy) and multiclass (12 classes) classification tasks using specific, total, and mixture models to achieve an accuracy of 97.47%, 70.08%, and 94.7% for specific, mixture, and total specific models for the identification of cancer. Owais et al. [144] deployed a DL-based classification framework for the diagnosis of gastrointestinal diseases from endoscopic images. They deployed two datasets that are publicly available: Kvasir dataset and Gastrolab dataset. They followed a 2-step process. The classification network predicts the disease type in the first step, and then in the second step, the retrieval part shows the relevant cases. They performed multiclass (37 classes) classification using DenseNet transfer learning architecture, LSTM architecture, PCA, and KNN methods to achieve a correct recognition rate of 96.19% on this task. The authors in [145] proposed a CNN-based DL architecture for the multiclass (4 classes) classification of acute lymphoblastic leukemia. They used stained bone marrow images achieving an accuracy of 97.78%. Kann et al. [146] deployed a 3D CNN model to identify nodal metastasis and tumor extranodal extension. Their dataset has 2875 CT samples, 124 samples for validation and 131 samples for testing. They used a series of rotations and flipping technique to augment the datasets while achieving an AUC of 0.91. The authors in [147] proposed a DL approach to study the limited sample training problem from holographic images. They studied the classification of healthy and cancer cell lines. They used Generative Adversarial Networks (GANs) as the data augmentation method to train a large number of unclassified samples from sperm cells. Their model achieved an accuracy of 99% for healthy/primary cancer/metastatic cancer multiclass classification problems.

Table 5 displays a summary of the studies for the task of classification of cancers covered in this subsection.

### 4.5. Classification, Segmentation, Prediction, and Detection of Brain Tumors

Sun et al. [148] proposed a 3D fully convolutional network-based multipathway architecture to extract features from MRI images from the BRATS 2019 challenge for the segmentation of brain tumor regions. They used the concept of dilated convolutions in each pathway to achieve a dice score of 0.89, 0.78, and 0.76 for whole tumor (WT), tumor core (TC), and enhancing tumor (ET) on the BRATS 2019 challenge, respectively. They used cropping, random slicing, and *z*-score normalization as the preprocessing methods. The authors in [149] proposed a novel architecture combining U-Net encoding and decoding subarchitecture, dilated convolutional feature extracting layers, and a residual module. Their proposed architecture achieved a dice score of 0.843, 0.897, and 0.906 and 0.798, 0.902, and 0.845 on ET, WT, and TC brain tumor subregions on BRATS 2018 and BRATS 2019 challenges, respectively. They used normalization and cropping techniques to preprocess the images. Khan et al. [150] utilized VGG16 and VGG19 transfer learning-based CNN models, partial least square covariance matrix, discrete cosine transform, and extreme learning machine to extract and classify features on BRATS 2015, BRATS 2017, and BRATS 2018 challenge datasets to achieve an accuracy of 97.8%, 96.9%, and 92.5% for BRATS 2015, BRATS 2017, and BRATS 2018 datasets, respectively. To preprocess the images before feeding them to the classification model, the authors used the histogram equalization approach. Pei et al. [151] proposed a joint deep and machine learning-based model for classification, segmentation, and prediction of brain tumors. Using a context-aware CNN architecture for segmentation, 3D CNN architecture for classification, and LASSO for prediction, the authors achieved a dice score of 0.821, 0.895, and 0.835 for ET, WT, and TC regions, respectively, on BRATS 2019 for the segmentation task, an accuracy of 58.6% for the survival prediction task on the BRATS 2019 dataset, and balanced accuracy of 63.9% on the test set for the 2019 Computational Precision Medicine Radiology-Pathology (2019 CPM-RadPath) challenge. The authors in [152] proposed a resource-efficient CNN model integrating memory connections and an adaptive dense block for the segmentation of brain tumors. They used the BRATS 2015 challenge dataset for the validation of their model and *z*-score normalization as a preprocessing method achieving a dice coefficient score of 0.858, 0.816, and 0.818 for WT, TC, and ET subregions. Badža and Barjaktarović [153] present a 22-layered CNN architecture for brain tumor classification of T1-weighted MRI images belonging to three categories: meningioma, glioma, and pituitary tumor. They normalize and resize the scans to 256 × 256 pixels followed by 90° rotation and vertical flipping augmentation methods to synthetically increase the size of the dataset. The authors achieved an accuracy of 96.56% for the multiclass classification task on a custom dataset. The authors in [154] proposed a transfer learning-based approach for segmentation and classification of brain tumors using Inception version 3-based features. They concatenated the CNN-based features with local binary pattern- (LBP-) based features. Contrast improvement is used as a preprocessing method. The authors achieved a dice score of 0.8373, 0.937, and 0.7994 for TC, WT, and ET subregions on the BRATS 2017 dataset and a dice score of 0.8834, 0.912, and 0.8184 for TC, WT, and ET subregions on the BRATS 2018 dataset. For the classification task, the authors achieved an average accuracy upward of 92% on BRATS 2013, BRATS 2014, BRATS 2017, and BRATS 2018 datasets. Rai et al. [155] proposed a U-Net-based DL model using skip connections for the classification, segmentation, and detection of tumors in brain MRI scans. They conducted their experiments on 120 patients of lower-grade glioma in TCGA database with 1373 scans for patients and 2556 scans for normal controls. The authors deployed cropping, resizing, global pixel normalization, horizontal flipping, flipping and rotation, random rotation, shift scale rotate, transposition, blurring, Gaussian blurring, random gamma, random brightness, and normalization as preprocessing and data augmentation methods. Their model achieved an accuracy of 99.7% on the classification task, a dice score of 0.9573 on the segmentation task, and a Jaccard index of 0.86 on the detection task. The authors in [156] compared and contrasted the performance of different transfer learning architectures for the binary classification of brain tumors into benign and malignant categories. They chose AlexNet, GoogLeNet, ResNet-50, ResNet-101, and SqueezeNet architectures for comparison. They employed a dataset of 224 benign category and 472 malignant category T1-weighted MRI images acquired from the TCIA public access repository. They used resizing, flipping, mirroring, salt noise addition, and rotation as preprocessing and data augmentation methods to achieve an accuracy of 99.04% using an AlexNet-type architecture. Feng et al. [157] developed a 3D U-Net model for brain tumor segmentation. They picked up an ensemble of models to extract features from brain MRI images on the BRATS 2018 challenge for segmentation and survival prediction. The authors achieved a dice score of (0.7946, 0.9114, and 0.8304) on (ET, WT, and TC) subregions for the segmentation task and an accuracy of 32.1% on the survival prediction task. The authors in [158] proposed an ensemble of deep CNN architectures integrating two and three paths of parallel models in a single model. They used 2D slices of brain MRI images from the BRATS 2013 dataset achieving a dice score of (0.86, 0.86, and 0.88) on (WT, TC, and ET) subregions. As a preprocessing step, they standardized the slices using the zero mean and unit variance normalization procedure. Naser and Deen [159] proposed a DL approach combining U-Net architecture, VGG16 transfer learning architecture, and a fully connected architecture for classification and segmentation of brain MRI images into lower-grade gliomas belonging to 110 patients. They used normalization, cropping, resizing, padding, rescaling, rotation, zooming, shifting, shearing, and flipping as preprocessing and data augmentation methods. Their approach achieved a dice score of 0.84 on the segmentation task and accuracy, sensitivity, and specificity of 92% on the binary classification (grade II/grade III) task. The authors in [160] proposed a multiscale 3D CNN architecture for the recognition and segmentation of 220 high- and 54 low-grade glioma MRI scans from the BRATS 2015 challenge dataset. As a preprocessing method, the authors used histogram matching to ensure consistency among gray levels. Their model achieved a dice score of 0.89 on the segmentation task, a sensitivity of 0.89, and a specificity of 0.90 on the recognition task. Chang et al. [161] proposed a DL model combining average pooling and max pooling layers along with 1 × 1 kernels. They further combined this model with conditional random fields to optimize prediction results. The authors used the BRATS 2013 dataset to achieve a dice score of (0.80, 0.75, and 0.71) on (WT, TC, and ET) subregions. As a preprocessing method, the authors used an intensity normalization method. The authors in [162] proposed a multiscale CNN model for the categorization of an MRI scan into healthy, meningioma, glioma, and pituitary tumor categories. The authors used 2D MRI images acquired from local hospitals in China to conduct their experiments. They achieved a dice score of (0.894, 0.779, 0.813, and 0.828) on (meningioma, glioma, pituitary tumor, and average), respectively, and accuracy of 97.3% on the classification task. As preprocessing and data augmentation methods, the authors used pixel standardization and elastic transformation methods.

Table 6 displays a summary of the studies for the classification, segmentation, prediction, and detection of brain tumors covered in this subsection.

## 5. Discussion

The dynamics of cancer growth with respect to time are difficult to estimate. Precise measures can be made largely at the end of the cycle in cancer's evolution, when it is detached from the body. Ongoing mutations provide a rich history of clonal lineages which lead to changes in both genotype and phenotype.

Psycho-oncology is a branch of oncology that deals directly with psychological and social issues. It deals with both emotional and psychobiological dimensions of cancer. However, there are still a number of obstacles in its wide adoption such as the dearth of medical practitioners as well as assessment tools and supporting instruments. It is important that both psychological and psychobiological factors influence the way cancers are treated. This domain must fulfill the demands for the availability of resources, support for caregivers and patients, and carving out new research directions for enthusiastic researchers [163, 164].

Research in AI has proven its worth in the support of medical decision-making. Due to the unknown nature of these algorithms, their widespread adoption is still limited. Explanatory AI algorithms provide a solution to this problem. However, performance issues might hinder their adoption as well. Robustness, local attribution, and completeness are three key properties of an explainable AI system. One way to get around this problem is to find strategies that optimally merge explainable and nonexplainable AI models. Some solutions that point in this direction are winning the confidence of clinicians by marking the regions in an image that are involved in AI predictions; another way is to attack or deceive the DL models through adversarial augmentations as it could potentially reveal the important features and discard the unimportant ones. There is a close link between interpretability and explainability. An explainable model is interpretable, but the reverse connection may not hold. A prediction relying on thousands of parameters is neither interpretable nor explainable [165, 166].

Precise DL model predictions are dependent on the availability of a large corpus of data (labelled or unlabelled), and it is a challenge to train it on a relatively small dataset. One way to look at this problem is through understanding the genetic evolution process. Gene transfer is the transfer of genetic information from a parent to its offspring. Genes encode genetic instructions (knowledge) from ancestors to descendants. The ancestors do not necessarily have better knowledge; yet, the evolution of knowledge across generations promotes a better learning curve for the descendants. There is a need for methods that can mimic this behaviour and use a limited number of examples to achieve their desired performance on different tasks [167]. Catastrophic forgetting is another problem limiting the performance of modern networks as they lack the ability to learn from continuous streams of data. The quality of the feature representation considerably determines the amount of forgetting. Boosting secondary information is the key to improving the transferability of features from old to new tasks without forgetting and is a promising direction for future work [168] especially for cancer diagnosis, prognosis, and prediction.

Despite the claims made by researchers, multiclass classification is an immensely difficult problem requiring a deeper understanding of human visual perception that moves beyond large datasets, and DL is perhaps necessary to solve many domain problems [169] including cancer diagnosis, prognosis, and prediction.

Another challenge that is worth mentioning is to find intricate hierarchical patterns from all forms of data such as labelled and unlabelled in a way that integrates information to perform visual inference. Unsupervised and semisupervised learning can help in this direction by offering potential solutions that help us in delving deeper into cancer pathogenesis and prediction tasks [170].

Can we use real-world images from another domain for calibration? Bridging the gap between cross-domain calibration and in-domain calibration is required to get optimal performance from neural networks. Techniques such as gram matrix similarity can be used as a criterion to select calibration datasets from a candidate pool to further improve performance [171]. This process can be used for effective feature construction in cancer diagnosis, prognosis, and prediction.

Modern DL object detection networks rely heavily on region proposal calculating algorithms to identify object locations. However, region proposal computation is a slow task. Faster region CNNs solve this problem by sharing convolutional layers with object detection subsystems. This process requires further research, and there is a need for improved computationally lightweight methods [25, 26]. Cancer lesion detection can be improved by doing thorough research in this domain.

Modern DL networks rely heavily on global image statistics. This reliance can cause problems for these systems as shape and texture recognition is often better done at the local rather than the global level. Research in this domain can lead to better network generalization [172] holding the potential to improve cancer diagnosis, prognosis, and prediction.

Mitigating gradient explosion or decay in RNN training based on pondering over informative inputs to strengthen their contribution in the hidden state and finding computationally efficient ways for this purpose by suppressing noise in inputs or imposing novel constraints is a problem worth investigating [173].

Image recognition and image generation are two cornerstones of computer vision. While both are burgeoning fields, specialized techniques from both subareas can sometimes form a dichotomy. Historically, the field of DL was widely popularized in discriminative image classification with AlexNet architecture and image generation through GANs and Variational Autoencoders (VAEs). Novel data augmentation methods that force a network to pay attention to the moments extracted by layers of a deep network are a need of time [174] and can improve the performance of models in cancer diagnosis, prognosis, and prediction.

Further research should also target the discovery of novel objects (such as those having an aberrant organization, rare tumor, and foreign bodies), interpretable DL models (using influence functions or an attention mechanism), intraoperative decision-making, and tumor-infiltrating immune cell analysis. Some problems such as the appearance of whole-slide image as orderless texture-like image and color variation and artefacts are potentially hindering the performance of DL techniques [175] for cancer diagnosis, prognosis, and prediction.

Different types of imaging modalities like mammography, CT, MRI, and ultrasound have helped in the staging of cancer especially breast cancer. These systems have helped medical practitioners in the early identification of breast cancer [176]. For breast cancer, varying types of breast densities make masses very difficult to detect and classify in comparison to calcifications providing room for further research in this domain [177].

Other areas for potential research are scarcity of data, imbalanced datasets, missing data, and high dimensionality of patient data. Future work should be focused on testing and improving methods to achieve better performing DL models for cancer diagnosis, prognosis, and prediction tasks.

## 6. Conclusion

DL models have revolutionized the diagnosis and predictions of cancers. Data have been accepted in various forms and multiple sources. These models are excellent feature extractors, and their characteristics can improve cancer prognosis and prediction. Data augmentation is important for cancer diagnosis and prediction tasks to improve the final performance of systems. These methods will play a key role in making predictions about the cancer diagnosis and prediction tasks. However, further testing and validation are required on larger datasets for clinical applications. More research on data augmentation methods, learning in different domains such as frequency domain, and deploying novel architectures such as graph convolutional networks will likely improve their performance further.

## Figures and Tables

**Figure 1:** Histopathological images of different cancer subtypes: (a) breast cancer, (b) skin cancer, (c) head and neck cancer, (d) brain cancer, (e) liver cancer, (f) colorectal cancer, (g) ovarian cancer, (h) lung cancer, (i) bladder cancer, (j) gastric cancer, (k) prostate cancer, and (l) pancreatic cancer.

**Table 1:** Summary of the datasets for cancer research.

Dataset/service/project	Link	Type(s) of cancer(s)	Description
TCGA database	https://www.cancer.gov/aboutnci/organization/ccg/research/structural-genomics/tcga	Multiple	33 cancer types, total no. of cases is 11125
Rotterdam tumor bank	https://stat.ethz.ch/R-manual/R-devel/library/survival/html/rotterdam.html	Breast cancer	2982 primary breast cancer patients; 1546 are positive cases
SUPPORT database	[31]	Multiple	9105 adults, an overall 6-month mortality rate of 47%
METABRIC dataset	https://www.cbioportal.org/study/summary?id=brca_metabric	Breast cancer	2509 primary breast tumor subjects, 548 matched normal control subjects
MITOS-ATYPIA-14 dataset	https://mitos-atypia-14.grand-challenge.org/Home/	Breast cancer	Resolution of 1539 × 1376 pixels at 20x and 40x magnification levels
TUPAC 2016 dataset	[33]	Breast cancer	500 training and 321 testing breast cancer histology whole-brain slides
INbreast dataset	[34]	Breast cancer	Total of 115 cases and 410 images
LIDC-IDRI database	https://wiki.cancerimagingarchive.net/display/Public/LIDCIDRI#1966254194132fe653e4a7db00715f6f775c012	Lung cancer	CT scans of 1018 subjects, three categories (i) nodule ≥ 3 mm, (ii) nodule < 3 mm, and (iii) nonnodule ≥ 3 mm
LUNA16 dataset	https://luna16.grandchallenge.org/Data/	Lung cancer	888 CT scans, facilitates segmentation studies
BreakHis dataset	https://web.inf.ufpr.br/vri/databases/breast-cancerhistopathological-database-breakhis/	Breast cancer	9109 microscopic images; four different magnification levels which are 40x, 100x, 200x, and 400x collected from 82 subjects
2015 Bioimaging Breast Histology Classification Challenge	https://rdm.inesctec.pt/dataset/nis-2017-003	Breast cancer	Four classes which are normal, benign, in situ carcinoma, and invasive carcinoma; resolution of 2040 × 1536 pixels
CAMELYON dataset	https://camelyon17.grand-challenge.org	Breast cancer	Facilitates patient-level analysis; 1399 unique whole-slide images; no metastases, macrometastases, micrometastases, and isolated tumor cells
PatchCamelyon dataset	https://www.tensorflow.org/datasets/catalog/patch_camelyon	Breast cancer	327,680 color images with resolution of 96 × 96 pixels; bigger than CIFAR10 and smaller than ImageNet dataset
2018 ICIAR dataset	https://iciar2018-challenge.grand-challenge.org/Dataset/	Breast cancer	Represent normal, benign, in situ carcinoma, and invasive carcinoma; 400 microscopy images with 100 images per class
MITOS12 dataset	http://ludo17.free.fr/mitos_2012/dataset.html	Breast cancer	50 biopsy slides; 40x magnification level; more than 300 mitoses
Leukemia microarray gene data	https://www.bioconductor.org/packages/devel/data/experiment/manuals/leukemiasEset/man/leukemiasEset.pdf	Bone marrow cancer	60 bone marrow samples; acute lymphoblastic leukemia, acute myeloid leukemia, chronic lymphocytic leukemia, chronic myeloid leukemia, and healthy bone marrow
Gene Expression Omnibus repository	https://www.ncbi.nlm.nih.gov/geo/	Multiple	Provides comprehensive sets of microarray, next-generation sequencing, and other genomic data
BioGPS data portal	http://biogps.org/#goto=welcome	Multiple	Supports eight species including humans; supports different types of cancers
TCIA	https://www.cancerimagingarchive.net	Multiple	Supports a large number of modalities; supports data such as patient outcomes, treatment details, and genomics
GDC	https://gdc.cancer.gov	Multiple	Provides genomic, clinical, and biospecimen data
TARGET	https://ocg.cancer.gov/programs/target#	Multiple	Childhood cancers are supported; provides vast amounts of genomic data to estimate molecular alterations
1000 Genomes Project	https://www.internationalgenome.org/1000-genomes-summary	Multiple	Provides a comprehensive resource on human genetic variation
Kvasir dataset	https://dl.acm.org/do/10.1145/3193289/abs/	Gastrointestinal tract cancer	4000 annotated images belonging to 8 classes
UCSB-BB dataset	https://bioimage.ucsb.edu/research/bio-segmentation	Supports breast cancer research in human species	Contains images of human, monkey, and cat species at subcellular, cellular, and tissue levels
BRATS dataset	https://www.med.upenn.edu/cbica/brats2020/	Brain tumor	MRI scans of 65 subjects each in clinical and synthetic datasets, for brain tumor segmentation task

**Table 2:** Summary of the studies for the prognosis/prediction of cancers.

Publication	Type(s) of cancer	Type of data	Methods	Performance
[50]	Astrocytic tumor	Microarray gene dataset	ANN	96.15% accuracy
[51]	Breast cancer	Nuclear morphometric features	ANNs	Good (>5 years) and bad (<5 years) prognoses
[52]	Breast invasive carcinoma	Gene expression data	Multiomics neural networks	Improved performance using more omics data
[53]	Breast cancer	TCGA	Random forest, neural network	Log-rank *p* < 0.05
[54]	Malignant melanoma	Custom dataset	Nonlinear ANN model	ANN model performs better than Cox model
[55]	Multiple	WHAS, SUPPORT, METABRIC, Rotterdam tumor bank	Deep feedforward neural network	Better prognostic accuracy than the clinical experts for the prognosis of nasopharyngeal carcinoma
[56]	Glioblastoma multiforme	TCGA	Pathway-associated sparse deep neural network	AUC = 0.6622 ± 0.013, *F*_1_ = 0.3978 ± 0.016
[57]	Breast cancer	Gene expression profile+copy number alteration profile+clinical data	Multimodal deep neural network	The proposed method achieves better performance than the prediction methods with single-dimensional data and other existing approaches
[58]	Hepatocellular carcinoma	TCGA	DL-based model	*p* value = 7.13 × 10^−6^ Concordance index = 0.68
[59]	Colorectal cancer	Images of tumor tissue samples	Combined convolutional and recurrent architectures	Prediction with only small tissue areas (hazard ratio 2.3), tissue microarray spot (hazard ratio 1.67), and whole-slide level (hazard ratio 1.65)
[60]	Ovarian cancer	CT images	Combined DL and Cox proportional hazards model	Concordance index was 0.713 and 0.694
[61]	Multiple	TCGA	ANN framework	Same or better predictive accuracy compared to other methods
[62]	Multiple	WHAS, SUPPORT, & METABRIC	Cox proportional hazards deep neural network	Superior in predicting personalized treatment recommendations
[63]	Lower-grade glioma and glioblastoma	TCGA	CNNs	Median concordance index = 0.754
[64]	Mesothelioma	TCGA+French source	CNNs	Concordance index of 0.656 on TCGA cohort
[65]	Multiple	TCGA+Gene Expression Omnibus dataset	DL-based model	For both marker types, the specificity of normal whole blood was 100%

**Table 3:** Summary of the studies for the segmentation/detection of cancers.

Publication	Type(s) of cancer	Type of data	Methods	Performance
[66]	Breast cancer	Ultrasound images, 2 datasets (A & B)	LeNet, U-Net, AlexNet	*F*‐measure = 0.91 (on dataset A) and *F*‐measure = 0.89 (on dataset B)
[67]	Breast lesions	Two custom datasets	FCN-AlexNet, FCN-32s, FCN-16s, and FCN-8s	Dice score of 0.7626 (FCN-16s)
[68]	Breast cancer	Camelyon16	DL algorithm	Slide-level AUC of 99%
[69]	Breast cancer	International Conference on Pattern Recognition 2012, MITOS-ATYPIA-14, Tumor Proliferation Assessment Challenge 2016	Faster region CNN, ResNET-50, DenseNet-201	0.691 *F*_1_-measure for the MITOS-ATYPIA-14 dataset
[70]	Multiple	Custom histopathology image dataset	Multilayer perceptron, logistic modal tree, sequential minimal optimization, Naïve Bayes, random forest, rotation forest, J-Rip, and PART algorithms	Rotation forest algorithm achieved an accuracy of 85.7% for binary classification between cancerous and noncancerous cells
[71]	Breast cancer	ICPR 2014 mitosis dataset, TUPAC 2016 mitotic cell dataset	Modified regional CNN	Precision = 0.76, recall = 0.72, *F*_1_‐score = 0.736 on TUPAC 2016 dataset
[72]	Breast cancer	Custom dynamic contrast-enhanced MRI dataset	3D deep CNN architecture	83.7% accuracy, 90.8% sensitivity, 69.3% specificity, AUC of 0.859, overall dice distance of 0.501 ± 0.274
[73]	Breast cancer	INbreast database	Different DL methods	Accuracy of 98.96%, MCC of 97.62%, *F*_1_-score of 99.24%, Jaccard similarity coefficient of 86.37%
[74]	Lung nodules	LUNA16, LIDC-IDRI	Two deep 3D customized mixed link network encoder-decoder architectures	Accuracy of 94.17%
[75]	Lung cancer	LIDC-IDRI dataset, Kaggle data science bowl challenge dataset	3D CNN architectures	Dice coefficient for LIDC-IDRI of 0.40, with 0.25 precision and 0.93 recall
[76]	Bladder cancer	Custom datasets	DL algorithm	Per-frame sensitivity and specificity were 90.9% and 98.6%
[77]	Full body	PET images	DL-based approach	Dice score of 0.93 ± 0.05
[78]	Brain metastases	Custom MRI dataset	DL-based approach (faster region-based CNN model)	96% sensitivity, AUC = 0.79
[79]	Thyroid nodules	Two custom datasets of ultrasound images	You only look once v3 dense multireceptive field CNN	mAP = 90.05 and 95.23
[80]	Liver cancer	225 CT scans of hemangioma, hepatocellular carcinoma, and metastatic carcinoma	Watershed segmentation, Gaussian mixture model (GMM), and deep neural network	Dice score of 0.9743, accuracy of 99.38%
[81]	Liver cancer	KMC liver dataset, multiorgan Kumar dataset	DL model combining residual block, bottleneck block, and attention decoder	Jaccard index of 0.7206 on KMC liver dataset and 0.6888 on Kumar dataset
[82]	Colorectal cancer	MICCAI gland segmentation dataset, colorectal adenocarcinoma gland dataset	Modified U-Net-based architecture	Dice score of 0.929 on MICCAI gland segmentation dataset, 0.89 on the colorectal adenocarcinoma gland dataset
[83]	Colorectal cancer	Custom dataset of MRI images of 28 adenocarcinomas and 5 mucinous carcinomas	CNN architecture which is a combination of three CNN architectures	Dice score of 0.60, precision of 0.76, and recall of 0.55
[84]	Ovarian cancer	Custom dataset of 127 patients and a total of 469 images	U-Net models	Dice score of 0.87, an average Pearson correlation of 0.90, and an average intraclass correlation of 0.89
[85]	Gastric cancer	Custom dataset of 1208 healthy and 533 endoscopic images	Mask R-CNN algorithm	Average dice index of 71%
[86]	Gastric cancer	Custom dataset of 1340 pathological slices	Deeplab v3+	Dice score of 0.9166
[87]	Prostate cancer	MRI images from an online database	DL system combining four U-Net models	Overall average accuracy of 95.3%
[88]	Prostate cancer	Custom dataset of 1200 ultrasound images	DL method integrating mask R-CNN and Inception version 3 models	Dice score of 0.88, a precision of 76% on malignant and 75% on benign classes for the classification task using an Inception v3 architecture
[89]	Prostate cancer	Custom dataset of CT images of 556 cases	2D U-Net model	Dice score of 0.85, 0.94, and 0.85 for prostate, bladder, and rectum, respectively
[90]	Pancreatic cancer	Custom dataset of T1w MRI images of 40 subjects	CNN architecture	Dice score of 0.73
[91]	Pancreatic cancer	Custom dataset of MRI images belonging to 73 patients	DL method using spiral transformation	Dice score of 0.656 ± 0.1021

**Table 4:** Summary of the studies for the classification of breast cancer.

Publication	Type of data	Methods	Performance
[92]	Custom dataset of ultrasound images	Pretrained CNNs	AUC of 0.90 (nonmalignant vs. malignant), AUC of 0.88 (benign vs. malignant)
[93]	1 custom+2 publically available datasets	DL-based approach using a matching layer	AUC = 0.936 (custom dataset), AUCs around 0.89 (publically available datasets)
[94]	Custom dataset of ultrasound images	Inception v3, VGG19	Robust and efficient classification performances
[95]	Custom dataset of ultrasound images	Training from scratch, pretrained VGG16, fine-tuning approach	0.97 accuracy, 0.98 AUC using fine-tuning approach
[96]	Custom dataset of breast MRI images	Cross-modal transfer learning approach	Overall accuracy of 0.93 using cross-modal approach
[97]	Custom dataset of breast MRI images	DL-based method	High sensitivity in the range of 93-100%
[98]	Custom dataset of multiparametric MRI images	Pretrained CNN architectures	AUC_feature fusion_ = 0.87
[99]	BreakHis, Breast Cancer Classification Challenge 2015	Inception recurrent residual CNN model	100% for the binary and multiclass (Breast Cancer Classification Challenge 2015 dataset)
[100]	BreakHis	Single-task CNN, multitask CNN	Patient score of 83.72% for binary classification using single-task CNN
[101]	2015 bioimaging breast histology classification challenge, BreakHis dataset	Progressive DL-based models	Recognition rate of 96.4% and 99.5% on multiclass and binary classification tasks on 2015 bioimaging breast histology classification challenge
[102]	BreakHis dataset, PatchCamelyon dataset, 2015 Bioimaging challenge dataset, 2018 ICIAR dataset	VGG19, MobileNet, DenseNet	Accuracy of 98.13% on BreakHis dataset
[103]	BreakHis dataset	DL and hierarchical classification approach	Accuracy of 95.48% on the multiclass classification task
[104]	BreakHis dataset	Integrated DL model	98.51% classification success on the multiclass classification task
[105]	BreakHis dataset	DenseNet and Xception architectures	99% and 92% accuracy on binary and multiclass classification tasks
[106]	BreakHis dataset	DL-based model	Mean recognition rate of 90.0 ± 6.7 for binary classification
[107]	BreakHis dataset	DL-based model	Accuracy of 94.7 ± 3.6 for multiclass classification
[108]	BreakHis dataset	Bag of words, locality-constrained linear coding, CNNs	For CNN model accuracies between 96.15% and 98.33% for the binary classification and 83.31% and 88.23% for the multiclass classification
[109]	BreakHis dataset	Combination of 4 residual networks	Correct classification rate of 96.25% for 8-class categorization
[110]	BreakHis dataset	End-to-end model based on FCN and bidirectional LSTM	Accuracy of 96.32 ± 0.51 on binary classification task
[111]	BreakHis dataset	ResNet-18, ResNet-50, and AlexNet	Image-level accuracy of 96.88% for binary classification
[112]	BreakHis dataset	Weakly supervised learning framework	Classification rate of up to 92.1% for binary classification
[38]	2015 Bioimaging challenge dataset	CNN models	Accuracies of 77.8% for four classes and 83.3% for carcinoma/noncarcinoma were achieved
[113]	ICIAR 2018 Grand Challenge	Pretrained ResNet-50, Inception v3, and VGG16 architectures	Accuracies of 87.2% for multiclass, 93.8% for binary classification tasks
[114]	2015 Bioimaging challenge database	Clustering algorithm and ResNet-50 architecture	88.89% accuracy on the overall test set for multiclass classification
[115]	BreakHis dataset	VGG16, VGG19, and ResNet-50 architectures	92.60% accuracy
[116]	Custom dataset	CNN, KNN, Inception v3, SVM, and ANN models	Accuracy of 97% using ANN algorithm for binary classification
[117]	Custom dataset	CNN and ANN models	Accuracy of 92.02 ± 0.51% for the binary classification task using a VGG model, accuracy of 92.02 ± 0.48% for the multiclass classification task
[118]	BreakHis dataset	VGG16, VGG19, ResNet-50 architectures	Accuracy of 93.25% for multiclass classification task
[119]	BreakHis dataset	DL-based model	*F*_1_-score of 90.3
[120]	BreakHis dataset	Deep second-order pooling network	Accuracy of 97.92% for binary classification
[121]	BreakHis+custom datasets	Pretrained CNN architectures (GoogLeNet, VGGNet, and ResNet)	Accuracy of 97.67% for binary classification
[122]	Custom dataset	Transformer models	Precision of 0.976 for relation recognition
[123]	Australian Breast Cancer Tissue Bank, TCGA dataset	Deep neural network	AUC on TCGA of 0.861, AUC on Australian Breast Cancer Tissue Bank was 0.905
[124]	INbreast database	DL models	AUC = 0.98

**Table 5:** Summary of the studies for the classification of other types of cancer.

Publication	Type(s) of cancer	Type of data	Methods	Performance
[125]	Colorectal cancer	Custom dataset	VGG19, AlexNet, SqueezeNet version 1.1, GoogLeNet, ResNet-50	98.7% accuracy using VGG19 model
[126]	Colon cancer	Custom dataset	CNN model	AUC = 0.998, specificity = 99.7%, sensitivity = 100%
[127]	Gastric cancer	Custom datasets	DL models	Accuracy of 0.822 in the international validation cohort
[128]	Bladder cancer	TCGA+custom dataset	DL models	Accuracy (custom) = 75%
[129]	Lung cancer	TCGA+custom dataset	Weakly supervised DL algorithm	Accuracy of 97.3% on the custom dataset
[130]	Prostate cancer	Custom dataset	DL methods	Accuracy of 92% in cancerous/benign classification
[131]	Skin cancer	Custom dataset	DL algorithms	Positive predictive value of 59.9%
[132]	Skin cancer	HAM10000, Kaohsiung Chang Gung Memorial Hospital	Lightweight DL algorithm	Accuracy = 85.8% (HAM10000, multiclass classification)
[133]	Skin cancer	Custom dataset	Interpretable DL methods	Accuracies between 93.6% and 97.9%
[134]	Skin cancer	Custom dataset	CNN model	Accuracy of 82.95% for multiclass classification
[135]	Liver cancer	TCGA dataset	DL model	High accuracy (abnormal/normal classification)
[136]	Head and neck cancer	Custom dataset	Inception version 3	Mean AUC was 0.936 based on the testing set
[137]	Pancreatic cancer	Three custom datasets	CNN architectures	Accuracy of 0.986 for test set 2
[138]	Multiple	Custom datasets	ResNet-18, ResNet-34, ResNet-50	Accuracy of 94.90% for ResNet-50 architecture
[139]	Breast cancer	MITOS12, 2016 Tumor Proliferation Assessment Challenge	CNN architecture	*F*-measure of 0.79
[140]	Multiple	Custom dataset	Multiple instance learning-based DL system	Sensitivity = 100%
[141]	Blood and bone marrow cancer	Leukemia microarray gene data, Gene Expression Omnibus repository	Single-layer neural network, 3-layered deep network	96.67% for 3 layered model
[142]	Multiple	BioGPS data portal, TCIA, GDC dataset	Regression-based partitioned DL algorithm	Accuracy = 94.5%
[143]	Multiple	TCGA, 1000 Genomes Project	DL algorithms	Accuracy = 97.47%
[144]	Multiple	Kvasir dataset, Gastrolab	DL-based classification network	Accuracy = 96.19%
[145]	Multiple	Custom datasets	CNN model	Accuracy = 97.78%
[146]	Multiple	Custom dataset	3D CNN model	AUC = 0.91
[147]	Multiple	Custom dataset	GAN-based model	90–99% accuracies

**Table 6:** Summary of the studies for the classification, segmentation, prediction, and detection of brain tumors.

Publication	Dataset(s)	Task(s)	Method	Performance
[148]	BRATS 2019	Segmentation	3D fully convolutional network-based multipathway architecture	Dice score of 0.89, 0.78, and 0.76 for WT, TC, and ET subregions, respectively
[149]	BRATS 2018 and BRATS 2019	Segmentation	Combination of U-Net encoding and decoding subarchitecture, dilated convolutional feature extracting layers, and a residual module	Dice score of 0.843, 0.897, and 0.906 and 0.798, 0.902, and 0.845 on ET, WT, and TC brain tumor subregions on BRATS 2018 and BRATS 2019 challenges, respectively
[150]	BRATS 2015, BRATS 2017, and BRATS 2018	Classification	VGG16 and VGG19 transfer learning-based CNN models, partial least square covariance matrix, discrete cosine transform, and extreme learning machine	Accuracy of 97.8%, 96.9%, and 92.5% for BRATS 2015, BRATS 2017, and BRATS 2018 datasets, respectively
[151]	BRATS 2019 and 2019 CPM-RadPath	Classification, segmentation, and prediction	Context-aware CNN architecture for segmentation, 3D CNN architecture for classification, and LASSO for prediction	Dice score of 0.821, 0.895, and 0.835 for ET, WT, and TC regions, respectively, on BRATS 2019 for segmentation task, accuracy of 58.6% for survival prediction task on BRATS 2019 dataset, and balanced accuracy of 63.9% on 2019 CPM-RadPath challenge
[152]	BRATS 2015	Segmentation	Resource-efficient CNN model with memory connections and an adaptive dense block	Dice coefficient score of 0.858, 0.816, and 0.818 for WT, TC, and ET subregions
[153]	Custom	Classification	22-layered CNN architecture	Accuracy of 96.56%
[154]	BRATS 2013, BRATS 2014, BRATS 2017, and BRATS 2018	Segmentation and classification	Inception version 3+LBP	Dice score of 0.8373, 0.937, and 0.7994 for TC, WT, and ET subregions on BRATS 2017; dice score of 0.8834, 0.912, and 0.8184 for TC, WT, and ET on BRATS 2018; average accuracy upward of 92% on BRATS 2013, BRATS 2014, BRATS 2017, and BRATS 2018 datasets
[155]	TCGA database	Classification, segmentation, and detection	U-Net-based DL model using skip connections	Accuracy of 99.7% on the classification task, dice score of 0.9573 on the segmentation task, and Jaccard index of 0.86 on the detection task
[156]	TCIA public access repository	Classification	AlexNet, GoogLeNet, ResNet-50, ResNet-101, and SqueezeNet	An accuracy of 99.04% using AlexNet-type architecture
[157]	BRATS 2018	Segmentation and prediction	3D U-Net model	Dice score of 0.7946, 0.9114, and 0.8304 on ET, WT, and TC, accuracy of 32.1%
[158]	BRATS 2013	Segmentation	Ensemble of deep CNN architectures	Dice score of 0.86, 0.86, and 0.88 on WT, TC, and ET
[159]	Custom	Segmentation and classification	U-Net architecture, VGG16 transfer learning architecture, and a fully connected architecture	Dice score of 0.84; accuracy, sensitivity, and specificity of 92% on the binary classification task
[160]	BRATS 2015	Segmentation and classification	Multiscale 3D CNN architecture	Dice score of 0.89, sensitivity of 0.89, and a specificity of 0.90
[161]	BRATS 2013	Segmentation	DL model combining average pooling and max pooling layers along with 1 × 1 kernels	Dice score of 0.80, 0.75, and 0.71 on WT, TC, and ET
[162]	Custom	Segmentation and classification	Multiscale Convolutional Neural Network	Dice score of 0.894, 0.779, 0.813, and 0.828 on meningioma, glioma, pituitary tumor, and average and an accuracy of 97.3%

## Data Availability

No data were used to support this study.
